# A study on expression level and nutritional status of IGFBP-2 after left neck anastomosis combined with placement of feeding nutritional applicators carrying ^(125)I particles in the treatment of esophageal cancer

This article has been retracted.

**DOI:** 10.3389/fonc.2022.1085305

**Published:** 2022-12-06

**Authors:** Zhiqiang Zhan, Jiaqi Mei, Xiangwu Zhou, Sicong Jiang, Daojing Li, Xuefeng Wang

**Affiliations:** ^1^ Department of Oncology, Jiangxi Pingxiang People’s Hospital, Pingxiang, China; ^2^ The first clinical medical college of Nanchang University, Nanchang, China; ^3^ Department of Thoracic Surgery, Medical College of Nanchang University, Nanchang, China; ^4^ Division of Thoracic and Endocrine Surgery, University Hospitals and University of Geneva, Geneva, Switzerland; ^5^ Department of Radiotherapy, Jiangxi Province Cancer hospital, Nanchang, China; ^6^ Department of Hepatobiliary Surgery, Xiantao First People’s Hospital Affiliated to Yangtze University, Xiantao, China

**Keywords:** esophageal cancer, left neck anastomosis, placement of feeding nutritional applicators carrying ^(125)I particles, human insulin-like growth factor binding protein-2, Nutritional Status, prognosis

## Abstract

**Background:**

To explore the changes and significance of the expression level and nutritional status of human insulin-like growth factor binding protein-2 (IGFBP2) after the treatment of esophageal cancer with left neck anastomosis combined with placement of feeding nutritional applicators carrying ^(125)I particles.

**Methods:**

A total of 110 patients with esophageal cancer (observation group: left neck anastomosis combined with placement of feeding nutritional applicators carrying ^(125)I particles) and 100 healthy people (control group) were enrolled at the same period. Then enzyme-linked immunosorbent assay (ELISA) was carried out to detect level of IGFBP-2. Lymphocyte count and serum albumin were measured by immune analyzer and automatic protein analyzer to evaluate nutritional status. Logistic regression analysis was used to analyze the relationship between serum IGFBP-2, nutritional status and prognosis of esophageal cancer after combined treatment.

**Results:**

The albumin, lymphocyte absolute value and PNI detection value of the control group were lower than those of the observation group 1 month after treatment, and the difference was statistically significant compared with the control group. The detection value of IGFBP-2 in early patients before and after treatment was lower than that in middle and late patients, and the detection values of albumin, lymphocyte absolute value and PNI were higher than those in middle and late patients, the differences were statistically significant. Serum IGFBP-2 level was negatively correlated with PNI, and albumin and lymphocyte absolute value were positively correlated with PNI. The detection value of IGFBP-2 in patients with good prognosis was significantly lower than that in patients with poor prognosis, and the detection values of albumin, lymphocyte absolute value and PNI were significantly higher than those in patients with poor prognosis. The AUC (0.887,95% CI: 0.799-0.975) of IGFBP-2, albumin, lymphocyte absolute value and PNI in predicting poor prognosis of esophageal cancer was the largest, and the sensitivity and specificity were 94.12% and 92.47%, respectively.

**Conclusions:**

Left neck anastomosis combined with ^(125)I particle application nutritional tube is helpful for the decrease of serum IGFBP-2 and the increase of various nutritional status indicators, which is beneficial for the improvement of the patient’s condition.

## Introduction

Esophageal cancer, a malignancy arising from the esophageal epithelium, is commonly manifested as dysphagia, foreign body sensation behind the breast bone, *etc.* in clinic, probably accompanied by weight loss, emaciation, hematemesis, and other symptoms. As the disease progresses, the trachea may be involved, thereby leading to hemoptysis, and the large blood vessels may be invaded, which will probably induce massive hemorrhage, shock and even death. Hence, measures should be actively taken to control the progression of esophageal cancer in patients (1, 2). As the medical technology advances, individualized comprehensive treatment has currently become the mode adopted by most esophageal cancer patients, in which targeted treatment measures are formulated in consideration of the patients’ physical fitness and specific conditions. Generally, surgical resection is a preferred treatment option for tumor patients. For esophageal cancer patients, left neck anastomosis is usually combined with tumor resection to rebuild the digestive tract and provide conditions for postoperative nutritional support (3). At present, placement of feeding nutritional applicators carrying ^(125)I particles is a relatively novel treatment method. It can simultaneously achieve close treatment and gastrointestinal nutrition support, that is, while removing residual tumor cells, it provides effective nutritional support for patients after esophageal cancer surgery and promotes postoperative rehabilitation (4).. Emerging as a novel treatment method, left neck anastomosis combined with the placement of feeding nutritional applicators carrying ^(125)I particles has rarely been clinically applied and researched. It has been found that human insulin-like growth factor binding protein-2 (IGFBP-2) participates in the occurrence and development of multiple malignancies, and this substance performs vital biological functions in the proliferation and migration of tumor cells by mediating dependent or independent IGF ligands (5). Malnutrition becomes a widely existing postoperative event in patients with esophageal cancer under the influences of such factors as the lesion site and postoperative treatment, which will have direct impacts on their immune function recovery and prognosis (6). In this study, therefore, the changes in the serum IGFBP-2 level and nutritional status in patients with esophageal cancer before and after left neck anastomosis combined with placement of feeding nutritional applicators carrying ^(125)I particles and in healthy people were compared and analyzed, so as to explore the roles of the serum IGFBP-2 level and nutritional status in the treatment of esophageal cancer with left neck anastomosis combined with placement of feeding nutritional applicators carrying ^(125)I particles.

## Patients and methods

### Patients

A total of 110 patients with esophageal cancer (observation group) admitted to our hospital and 100 healthy people undergoing physical examination in our hospital (control group) from January 2020 to December 2021 were selected as the research subjects.The basic data showed no statistically significant differences between the two groups (P*>*0.05), as shown in **Table 1**. The research subjects voluntarily signed the informed consent, and this study was approved by Jiangxi Pingxiang People’s Hospital Ethics Committee. The research program is in line with the Helsinki Declaration.

**Table 1:** The basic data of both groups.

	Gender (male)	Age (years)	BMI (kg/m2)	Education level		
				Middle school or below	Postsecondary specialized college	University
Observation group	66	(60.03 ± 6.95	22.97 ± 2.31	33	46	31
control group	69	60.51 ± 6.92	22.84 ± 2.27	28	45	27
t/χ2	0.244	0.5	0.411	0.221		
P	0.621	0.617	0.682	0.895		

BMI, Body Mass Index.

### Criteria for esophageal cancer screening

Symptoms such as dysphagia and retrosternal pain, the destruction of esophageal mucosa, stenosis of lumen, craters, and filling defects, as shown in Barium X-rays of the esophagus, positive esophageal exfoliated cells, and stenosis of the lumen and destruction of the mucosa, as shown in esophagoscopy, are suggestive of esophageal cancer (7).

### Inclusion and exclusion criteria

Inclusion criteria involved: 1) patients aged ≥18 years old, 2) those with complete basic data, and 3) those pathologically diagnosed with esophageal cancer. Exclusion criteria were shown below: 1) patients who had received radiotherapy or chemotherapy before inclusion, 2) those suffering from infectious diseases before inclusion, 3) those with other malignant tumors, 4) those with history of major surgery or trauma within 3 months before inclusion, 5) those complicated with immune system diseases or serious organic diseases, or 6) those who had participated in other experimental studies. Drop-out criteria were set below: 1) patients with mental disorder, language disorder, or low compliance, 2) those who dropped out of this research halfway, or 3) those who were lost to follow-up.

## Methods

### Test equipment and reagents

Test equipment and reagents included a high-speed cryogenic centrifuge (model: LXJ-II, Shanghai Medical Analysis Instrument Factory, Shanghai, China), a refrigerator for blood and plasma cryopreservation (Wuhan Hans Instrument & Equipment Co., Ltd., Wuhan, China), the enzyme-linked immunosorbent assay (ELISA) kit of IGFBP-2 and its accessories (Shanghai Enzyme-Linked Biotechnology Co., Ltd., Shanghai, China), a microplate reader (model: YT-SY96, Shandong Yuntang Intelligent Technology Co., Ltd., Weifang, China), an immunoassay analyzer (model: ST-MB96A, SANTIYIQI), an automatic protein analyzer (IMMAGE 800, Beckman Coulter, Franklin Lakes, NJ, USA), ^(125)I particles [Seeds Biological Pharmacy (Tianjin) Ltd., Tianjin, China], and a computed tomography (CT) scanner (model: Brilliance16, Philips).

### Indicator detection

The fasting elbow venous blood (5 mL) was collected from patients in observation group at admission and at 1 month after left neck anastomosis combined with placement of feeding nutritional applicators carrying ^(125)I particles, and from healthy people undergoing physical examination. After collection, the blood samples were placed in anticoagulation vacuum tubes, and centrifuged using a centrifuge at 15 cm×2000 r/min for 10 min. Then the obtained upper serum was stored in the refrigerator at -80. Later, the serum was taken out, placed at room temperature at 30 min before detection, and then subjected to routine procedures using the IGFBP-2 ELISA kit and the microplate reader. Specifically, 100 μL of the samples and standard substance were incubated at 37°C for 30 min to prepare solution, followed by washing. After that, the samples were incubated with 100 μL of avidin-horseradish peroxidase, and washed for 5 times. Next, 50 μL of developer A and 50 μL of developer B were added for 15-min color development away from light. Afterwards, 5 μL of stop solution was added for optical density determination using the microplate reader. Finally, the level of IGFBP-2 was detected. Meanwhile, the lymphocyte count and serum albumin level were measured using the immunoassay analyzer and automatic protein analyzer. Prognostic nutritional index (PNI) = peripheral blood lymphocyte count (× 10^9^) × 5 + serum albumin level (g/L).

### Treatment methods

All the patients in observation group underwent left neck anastomosis combined with placement of placement of feeding nutritional applicators carrying ^(125)I particles. The details were shown as follows.

Left neck anastomosis: Following combined intravenous-inhalation anesthesia, laparoscopic esophagectomy and left neck anastomosis were performed successively. A small incision was made at the anterior edge of the sternocleidomastoid muscle in the left neck, and dissociated to the esophagus and down to the top of the pleura. Then the cervical segment of the esophagus was dissociated, and the upper cervical segment of the esophagus was placed on an anastomotic staple holder, while the lower cervical segment of the esophagus was sutured with a traction band. Later, the esophagus and stomach were led out through the abdominal incision. The stomach was shaped like a tube with a linear cutting and closure device, and then the tubular stomach was lifted to the neck through the esophageal bed and anastomosed with the esophagus. Finally, the feeding jejunostomy tube and gastrointestinal decompression tube indwelled. After the operation, the wound was sutured.

Placement of feeding nutritional applicators carrying ^(125)I particles: ^(125)I particles were placed on an applicator equidistantly (5 mm) and attached to a nasal feeding nutritional tube, which was wrapped and fixed with surgical sutures. The patients were placed in the supine position and anesthetized locally with 2% lidocaine. Then a catheter and a guide wire were introduced from one nostril into the gastric cavity through the occluded esophageal segment, and a feeding nutritional applicator carrying ^(125)I particles was intubated along the guide wire to achieved CT-guided implantation of ^(125)I particles into the original tumor foci, followed by continuous low-dose radiation.

### Observational indicators

1) The IGFBP-2 level, albumin level, absolute lymphocyte count and PNI were compared. 2) In observation group, the IGFBP-2 level, albumin level, absolute lymphocyte count and PNI were compared between patients in tumor-node metastasis (TNM) stage I-II (early-to-middle stage) and those in TNM stage III-IV (middle-to-late stage). 3) The correlations of the serum IGFBP-2 level, albumin level and absolute lymphocyte count with PNI were analyzed. 4) IGFBP-2 level, albumin level, absolute lymphocyte count and PNI were compared between patients with good prognosis and those with poor prognosis in observation group. In addition, the patients in observation group were followed up for 6 months. The complete disappearance of tumor tissues after the combined therapy with no signs of recurrence indicated good prognosis, while the complete disappearance of tumor tissues after combined therapy with signs of tumor recurrence (including but not limited to the appearance of tumor at the original foci or new foci) indicated poor prognosis.

### Statistical analysis

Data were processed using Statistical Product and Service Solutions (SPSS) 25.0 software (IBM, Armonk, NY, USA). Count data were expressed as % and compared between groups using *χ^2^* test. Measurement data in line with the normal distribution were expressed by ( χ ± s), and independent samples *t* test was adopted for intergroup comparison, while the paired *t* test for intragroup comparison. Moreover, logistic regression analysis was carried out to investigate the correlations of the IGFBP-2 level, albumin level and absolute lymphocyte count with PNI. Besides, the receiver operating characteristic (ROC) curve was plotted to assess the application of the IGFBP-2 level, albumin level, absolute lymphocyte count and PNI in the prediction of prognosis. P<0.05 represented that the difference was statistically significant.

## Results

### Comparison of IGFBP-2, albumin, absolute lymphocytes, and PNI values

The IGFBP-2 detection value before treatment in the observation group was significantly higher than that 1 month after treatment in the observation group and the control group, while the albumin, absolute lymphocyte value and PNI detection value were lower than those 1 month after treatment in the observation group and the control group; the IGFBP-2 detection value 1 month after treatment in the observation group was lower than that before treatment, but still higher than that in the control group, and the albumin, absolute lymphocyte value and PNI detection value were higher than those before treatment, but still lower than that in the control group, and the differences had statistical significance (*P* < 0.05). See **Table 2**.

**Table 2:** Comparison of IGFBP-2, albumin, absolute lymphocytes, PNI values [x̅ ± s].

Group		Number of cases	IGFBP-2 (μg/L)	Albumin (g/L)	Absolute lymphocyte count (× 10 ^9^/L)	PNI
Observation group	Before treatment	110	301.83 ± 5.93 ^#^	31.94 ± 3.28 ^#^	1.57 ± 0.46 ^#^	39.79 ± 3.86 ^#^
	1 month after treatment	110	216.84 ± 5.38 ^*^	35.49 ± 3.61 ^*^	1.86 ± 0.62 ^*^	44.79 ± 4.03 ^*^
Control group		100	98.86 ± 4.29 ^#^	41.71 ± 3.96 ^#^	2.55 ± 0.68 ^#^	54.46 ± 4.82 ^#^
F-value		–	39000.120	194.520	75.230	321.700
P-value		–	< 0.001	< 0.001	< 0.001	< 0.001

^*^ P < 0.05 compared with pre-treatment and ^#^ P < 0.05 compared with 1 month post-treatment.

### Comparison of IGFBP-2, albumin, absolute lymphocyte and PNI values in patients with different TNM stages in the observation group

The IGFBP-2 values of patients in the middle and early stage before and after treatment were lower than those of patients in the middle and advanced stage, and the absolute values of albumin, lymphocytes and PNI values were higher than those of patients in the middle and advanced stage; compared with those before treatment, the IGFBP-2 values of patients in the middle and early stage and advanced stage esophageal cancer were significantly decreased, and the absolute values of albumin, lymphocytes and PNI values were increased, and the differences were statistically significant (*P* < 0.05). See **Table 3**.

**Table 3:** Comparison of IGFBP-2, albumin, absolute lymphocyte and PNI values in patients with different TNM stages [x̅ ± s].

Group		Number of cases	IGFBP-2 (μg/L)	Albumin (g/L)	Absolute lymphocyte count (× 10 ^9^/L)	PNI
Middle Early	Before treatment	62	293.76 ± 5.47	34.25 ± 3.51	1.79 ± 0.50	43.20 ± 3.98
	After treatment	62	209.38 ± 4.95	36.74 ± 3.77	2.03 ± 0.65	46.89 ± 4.12
t-Value _(Middle-Early Intragroup Comparisons)_		–	90.062	3.806	2.304	5.072
P-Value _(Middle-Early Intragroup Comparisons)_		–	< 0.001	< 0.001	0.023	< 0.001
Middle and advanced	Before treatment	48	312.25 ± 6.53	28.95 ± 2.98	1.29 ± 0.41	35.40 ± 3.71
	After treatment	48	226.48 ± 5.94	33.87 ± 3.40	1.64 ± 0.58	42.07 ± 3.91
t-Value _(Middle-late intragroup comparison)_		–	67.316	7.540	3.414	8.574
P-Value _(Middle-late intragroup comparison)_		–	< 0.001	< 0.001	0.001	< 0.001
t-value _(comparison between groups: pre-treatment)_		–	16.151	8.380	5.617	10.498
P-value _(between-group comparison: pretreatment)_		–	< 0.001	< 0.001	0.001	< 0.001
t-value _(comparison between groups: post-treatment)_		–	16.461	4.131	3.269	6.221
P-value _(between-group comparison: post-treatment)_		–	< 0.001	< 0.001	0.001	< 0.001

### Relationship analysis between serum IGFBP-2, albumin, absolute lymphocyte levels and PNI

Serum IGFBP-2 levels were negatively correlated with PNI, with higher IGFBP-2 values and lower PNI; absolute albumin and lymphocyte levels were positively correlated with PNI, with higher absolute albumin and lymphocyte values and higher PNI (*P* < 0.05). See **Table 4**.

**Table 4:** Relationship analysis between serum IGFBP-2, albumin, absolute lymphocyte levels and PNI.

Group	*β* value	*SE*	*Wald χ ^2^*	P-value	*OR*	95% CI
IGFBP-2	- 0. 212	0.007	9.171	0.0 23	0.810	0. 671 - 0.987
Albumin	0. 973	0.3 13	9.662	0.0 08	2.6 46	0. 958 -4. 281
Absolute lymphocyte count	0.9 68	0.3 12	9.624	0.01 2	2.6 33	0.9 46 -4. 086

### Comparison of IGFBP-2, albumin, absolute lymphocyte and PNI values in patients with different prognoses in the observation group

The IGFBP-2 values in patients with good prognosis were significantly lower than those in patients with poor prognosis, and the absolute values of albumin, lymphocytes and PNI values were significantly higher than those in patients with poor prognosis, and the differences were statistically significant (*P* < 0.05). See **Table 5**.

**Table 5:** Comparison of IGFBP-2, albumin, absolute lymphocyte and PNI values in patients with different prognoses in the observation group [x̅ ± s].

Group	Number of cases	IGFBP-2 (μg/L)	Albumin (g/L)	Absolute lymphocyte count (× 10 ^9^/L)	PNI
Favorable prognosis	93	113.02 ± 5.04	41.0 1 ± 3. 56	2.37 ± 0. 57	5 2.86 ± 4.13
Poor prognosis	17	287.85 ± 6.18	33.18 ± 3.19	1.25 ± 0.31	39.42 ± 3.50
t-value	–	126.862	8.46 3	7.871	12.603
P-value	–	< 0.001	< 0.001	< 0.001	< 0.001

Receiver operating characteristic (ROC) curves were plotted with prognostic effect as the independent variable (good prognosis = 0, poor prognosis = 1) and IGFBP-2, albumin, absolute lymphocyte value, and PNI level as the dependent variables, and the results showed that the AUC of IGFBP-2, albumin, absolute lymphocyte value, and PNI in combination with predicting poor prognosis of esophageal cancer (0.887, 95% CI: 0.799 – 0.975) was the largest, with sensitivity and specificity of 94.12% and 92.47%, respectively (*P* < 0.05). See **Table 6**.

**Table 6:** IGFBP-2, Absolute albumin, lymphocytes, PNI in poor prognosis of esophageal cancer.

Group	AUC	95% CI	Cut-off value	Sensitivity	Specificity	Youden index	P-value
IGFBP-2	0.678	0.581 to 0.775	> 251.04 μg/L	82.35	79.57	0.619	< 0.001
Albumin	0.602	0.509 to 0.695	< 35.00 g/L	70.59	72.04	0.426	< 0.001
Absolute lymphocyte count	0.592	0.506 to 0.678	< 2.11 × 10 ^9^/L	64.71	64.52	0.292	< 0.001
PNI	0.705	0.606 to 0.804	< 50.8	88.24	83.87	0.721	< 0.001
Combined	0.887	0.799-0.975		94.12	92.47	0.866	< 0.001

## Discussion

### IGFBP-2 in the combined treatment of esophageal cancer

Influenced by many factors such as our dietary preferences and dietary characteristics, the incidence rate and mortality rate of esophageal cancer in China are relatively high. Epidemiology shows that the incidence rate and mortality rate of esophageal cancer in China rank 6th and 4th among all malignant tumors respectively (8). With further research, it has been found that the occurrence of esophageal cancer is related to long-term smoking and alcohol consumption, poor dietary habits and excessive intake of nitrosamines, and that there is a certain genetic susceptibility to the development of esophageal cancer (9). Therefore, people with a family history of esophageal cancer, a love of pickled foods, long-term smoking and drinking, and excessive intake of irritating foods should pay attention to the prevention and treatment of esophageal cancer.

Left cervical anastomosis is a common surgical treatment for esophageal cancer. This treatment involves removing the tumour and at the same time moving the gastro-esophageal bed to the neck for anastomosis, so that patients can receive better nutritional support after surgery and achieve reconstruction of the digestive tract to solve their postoperative feeding problems (10). At the same time, when esophageal cancer is diagnosed, it is usually in the middle or late stage, and the tumor invades a large area. In this study, a left-sided cervical anastomosis was combined with a ^(125)I particle-loaded nutrition tube. This treatment combines nutritional support and chemotherapy treatment, with (125)I particles applied to the tube and covered by the tube, allowing the particles to radiate close to the original tumor lesion, effectively removing residual tumor cells around the original tumor lesion and further enhancing its overall anti-tumor therapeutic efficacy (11). In order to investigate the therapeutic effect of left-sided cervical anastomosis combined with ^(125)I particles in esophageal cancer, this study compared the IGFBP-2 expression level and nutritional status before and after treatment of esophageal cancer and in healthy physical examination patients at the same period. The IGFBP-2 detection values in the observation group before treatment were significantly higher than those in the observation group 1 month after treatment, and in the control group 1 month after treatment. The reasons for this are as follows: IGFBP-2 is a member of the insulin-like growth factor family, and this substance can affect the proliferation and migration of tumor cells by regulating chromatin structure and transcriptional sequences. In addition, IGFBP-2 has been found to regulate IGF and its integrin pathway, which can promote cell growth and proliferation (12). Based on this theory, in tumor diseases, high IGFBP-2 expression may promote the proliferation, growth and migration of tumor cells, which can promote tumor metastasis and aggravate the condition of patients. Michal et al. (13) et al. showed that serum IGFBP-2 assay values were higher in cancer patients compared to healthy subjects, and the survival rate was higher in those with high IGFBP-2 expression, which is consistent with the findings of this study. This indicates that changes in IGFBP-2 expression levels are related to changes in the condition of patients with esophageal cancer, and the significant decrease in IGFBP-2 test values in patients with esophageal cancer after combination therapy reflects that combination therapy can achieve significant therapeutic effects, and has a positive impact on controlling the development and improving the condition of patients with esophageal cancer.

### Nutritional status in the combined treatment of esophageal cancer

In terms of nutritional status, the results of this study showed that the albumin, lymphocyte absolute values and PNI test values of patients in the observation group before treatment were lower than those of the observation group one month after treatment and the control group; the albumin, lymphocyte absolute values and PNI test values of patients in the early and middle stage were higher than those of patients in the middle and late stage before and after treatment (P<0.05), suggesting that changes in nutritional status may be related to changes in the condition of patients with esophageal cancer. The reasons for this are analyzed as follows: the common clinical symptom of esophageal cancer is swallowing obstruction, and with the development of the disease, patients’ eating is significantly restricted. Compared with patients with other malignant tumours, malnutrition is more common and serious in esophageal cancer patients (14). The nutritional status is directly related to the immunity of the body. Lymphocytes and antibodies in the blood are made up of protein and other nutrients. The timely provision of nutritional support after surgery to improve the nutritional status of patients with esophageal cancer is of great significance in enhancing their immune function and promoting their post-operative recovery. Therefore, by measuring the absolute value of human lymphocytes and analyzing the level and production of lymphocytes, it can reflect the nutritional absorption of the patient. Although albumin does not directly enhance immunity, its physiological role includes maintaining intravascular colloid osmotic pressure, transport and detoxification, and participating in the immune response in the form of globulins. Keita et al. (15) showed that low expression of albumin was associated with worse disease and worse prognosis, which is consistent with the results of this study. The lower the absolute values of albumin, lymphocytes and PNI, the worse the nutritional status of the patient, and the more severe the disease.

The data of this study manifested that with regard to prognosis, the PNI was negatively correlated with the serum IGFBP-2 level but positively related to the albumin level and absolute lymphocyte count (P<0.05). Furthermore, the IGFBP-2 level was evidently lower, whereas the albumin level, absolute lymphocyte count and PNI were notably higher in patients with good prognosis than those with poor prognosis. Besides, the area under curve (AUC) [0.887, 95% confidence interval (95% CI): 0.799-0.975] of the combination of the IGFBP-2 level, albumin level, absolute lymphocyte count and PNI in predicting the poor prognosis of esophageal cancer patients was the largest, with the sensitivity and specificity of 94.12% and 92.47%, respectively (P<0.05). It can be seen that the changes of IGFBP-2 expression level and nutritional status may be related to the prognosis of patients with esophageal cancer. IGFBP-2 is a secreted protein, its synthesis and secretion are also related to the nutritional status of the body. Highly expressed IGFBP-2 can facilitate the proliferation and migration of tumor cells, intensify the invasion of tumor to surrounding normal tissues and organs, and then exacerbate symptoms such as dysphagia and retrosternal pain, thereby inducing and aggravating malnutrition. In this study, it was found that left neck anastomosis combined with placement of feeding nutritional applicators carrying ^(125)I particles effectively controlled and relieved esophageal cancer in patients, demonstrated by the removal of tumor tissues, a markedly decreased level of serum IGFBP-2, obviously relieved symptoms such as dysphagia, and the recovered nutritional absorption. At this time, the level of albumin and absolute lymphocyte count were on the rise.

## Conclusion

In summary, esophageal cancer patients exhibit a high expression of serum IGFBP-2, a low expression of albumin, a low absolute lymphocyte count and a low PNI. Therefore, the combination of serum IGFBP-2 level and nutritional status-related indicators (albumin level, absolute lymphocyte count and PNI) is more valuable in predicting the poor prognosis of esophageal carcinoma patients. The treatment of left neck anastomosis combined with ^(125)I particle application nutritional tube is helpful to the decrease of serum IGFBP-2 and the increase of various nutritional status indicators, which is beneficial to the improvement of the patient’s condition. Otherwise, the patient’s condition may deteriorate.But there were also some limitations, such as the sample of this retrospective study is small, weakening the evidence of the findings, thus should be further verified by future studies with large sample.

## Data availability statement

The original contributions presented in the study are included in the article/supplementary material. Further inquiries can be directed to the corresponding author.

## Ethics statement

The studies involving human participants were reviewed and approved by the ethics committee of Xiantao First People’s Hospital Affiliated to Yangtze University. The patients/participants provided their written informed consent to participate in this study.

## Author contributions

ZZ and XW designed the study and performed the experiments, JM and XZ collected the data, SJ and DL analyzed the data, ZZ and XW prepared the manuscript. All authors contributed to the article and approved the submitted version.
